The article "Design and Implementation of Smart Community Big Data Dynamic Analysis Model Based on Logistic Regression Model" was published in 2022. Journal: Comput Intell Neurosci.

# Design and Implementation of Smart Community Big Data Dynamic Analysis Model Based on Logistic Regression Model

**DOI:** 10.1155/2022/4038084

**Published:** 2022-06-22

**Authors:** Hong Jiang

**Affiliations:** ^1^College of Marxism, Shanghai University of Finance and Economics, Shanghai 200433, China; ^2^College of Marxism, Zhejiang Shuren University, Hangzhou 310015, Zhejiang, China

## Abstract

With the economic development, smart communities have been widely studied and applied. However, the system in this field is not perfect, and there are still a series of problems, such as high construction cost, low level of intelligence, mutual independence of different systems, difficulty in unified management, and so on. To solve the above problems, this paper proposes the smart community big data dynamic analysis model based on logistic regression model. First, this paper constructs the big data research architecture of smart community based on IOT technology, including IAAs, DAAS, PAAS, and SaaS layers and the virtual service layer of resource scheduling of spatiotemporal information cloud platform optimized by spatiotemporal law. And the IoT platform is designed to collect data to lay the foundation for research. Second, this paper is oriented to the big data application requirements with distribution and mobility as the main technical characteristics. Based on the distributed data flow, this paper designs mining operator to provide technical support for the data mining algorithm; at the same time, this paper constructs a high-dimensional random matrix model for measuring big data and then deduces its abnormal data detection theory and method to detect high-dimensional abnormal data. Finally, this paper uses logistic regression model to predict the development trend of smart community and provide guarantee for smart community service. The simulation results show the efficiency and accuracy of prediction can be improved based on logistic regression model. Furthermore, it effectively avoid repeated construction and waste of resources in the community and form a new community management model based on intelligent and information-based social management and service.

## 1. Introduction

With the economic development and the improvement of living standards, people's pursuit of living conditions no longer stays at the material level such as location, area, and price [1]. More attention is paid to the factors, such as community property, service, environment, and management. The traditional community construction and development model is difficult to continue [2]. At present, there is an urgent need for a new and effective community management and service system. Smart community refers to an intelligent and information-based ecological community built [3]. It has the characteristics of openness, comfort, and convenience. The concept of community information construction has been widely recognized and has become the general trend of residential community construction in the future [4]. Residential community is the product of social reform and the renewal of the living concept of urban and rural people. The development of the times and the progress of technology are bound to promote the continuous renewal of people's concept of living environment. Relying on IoT development, the smart community integrates the intelligent interconnection of each independent unit of the community and the home digital terminal into a comprehensive smart system, so that residents, property, and security personnel can exchange information, observe data, and provide real time and comprehensive services for community management. Since 2009, the IoT has been gradually widely used in many fields, such as urban safety, enterprise management, and convenient travel, and its market scale and economic benefits have exceeded trillions [5]. The Internet of things uses the terminal digital devices and sensors in the network to collect and upload data in real time, issue control instructions to realize the control of network monitoring entities, and finally form a huge network combined with the Internet [6]. Its purpose is to provide a network communication mode between things and people for human social behavior, so that equipment and tools have a sense of breathing. The development of domestic IoT technology also affects the development of key technologies in smart community systems such as sensor, wireless network, and label recognition, which provides technical support for the construction of smart communities [7].

Compared with the traditional mining methods, the classification mining of this kind of big data implies many challenging problems [8, 9]. First, the traditional classification mining method is based on a single learning sample set, and the distributed collection characteristics of big data determine that classification learning needs to be distributed; Second, the dynamic streaming big data are significantly different from the static data stored in the traditional database. It is impossible to store all the data at one time and then conduct offline mining [10]. We must explore the online real-time collection technology and the incremental mining method that changes with time; finally, the traditional classification mining technology has high requirements for the learning sample set, while the classification mining requires multinode and multistep collaborative processing [11]. Therefore, we must explore the classification technology with good performance according to the mining characteristics of this kind of big data, for this kind of distributed data collection and data streaming aggregation over time, the problem of classification mining in big data needs integrated technology and innovative theories and methods [12]. However, with the increasingly clear scientific problems, there have been some discussions on relevant mining frameworks and methods in recent years. Literature [x] proposed a distributed data stream mining algorithm DS means [13]. Its mining work is divided into three key steps: local clustering, pattern transmission, and global clustering. In order to adapt to the global fluctuation of data flow, the typical ds-means clustering algorithm is used in different time levels of distributed data flow. Before global node clustering, the number of global clusters is dynamically adjusted according to the clustering results of local nodes [14]. Literature [15] designs a distributed data evaluation algorithm ankle for multiple data streams, which solves the problem of parallel detection of data distribution changes by multiple nodes. Literature [16] constructs a distributed multinode mining framework for mining frequent item sets of distributed data streams to realize the key operation of the architecture.

Aiming at the common problems in the smart community, such as the independence of business systems, the inability to share resources, and the difficulty of unified management, this paper constructs a smart community management system based on IOT. Based on the logistic regression model, the cell resources and development trend are predicted, and the simulation results verify the reliability and effectiveness of the scheme.

## 2. Intelligent Community Architecture Design Based on IoT

### 2.1. Overall Structure Design of Smart Community System

The smart community system architecture is supported by information security and standard system, based on the IoT, and supported by urban public information platform and urban public basic database, has built a smart community comprehensive information service platform, and built a smart community comprehensive service application system for communities, owners, property, and enterprises, covering community interaction, property management, medical and health care, smart home, and smart community [17]. For applications in many fields such as smart government and convenient services, the system architecture is shown in Figure 1.

(1) Community is an important place for people's life. The intellectualization of community brings great convenience to people's life and work. Therefore, the safety, intelligence, and convenience of community are also the inevitable trend of community development. The demand of smart community is mainly reflected in the smart demand for home, property management, public services, and other aspects. Smart home has the characteristics of high security, convenient use, and cost saving. It can not only bring convenience to our life but also change our way of life; Smart Property Management covers business management informatization, all-in-one card management, comprehensive security, and equipment monitoring of property management department; Smart public service needs mainly include community portal, community medical care, elderly care, and one-stop window services; (2) the support platform is the basic function platform of the data centre integrating the construction of the data centre computer room, it infrastructure, cloud platform, and operation and maintenance management. It is the centre of the data storage and data circulation of the smart community system. It provides the operation environment for each application subsystem of the smart community, centrally manages the data, and completes the core functions such as hardware equipment construction, supporting software design, related product production, data management, and billing. The smart community public support platform provides strong data support for the upper application platform by building server equipment and integrates the data collected by each smart community into the platform. The supporting software development of the supporting platform adopts SOA (service-oriented architecture) architecture to design, provide the functions of service definition, development, deployment and operation, realize direct data communication between all layers, and realize the compatibility of modules between the same layers through service, so that the platform has good expansion ability. (3) In terms of network security construction of Hui community, it mainly provides safe and reliable community network for community residents by using information security technologies such as user identification, controlled access of terminal equipment, network firewall, and supporting antivirus software. At the same time, the security is strengthened through the management of segmented LAN, the excuse of data interaction, and the binding of network IP address.

Virtualization technology provides an effective solution for resource management in cloud computing model [18, 19]. By encapsulating services in virtual machines and mapping them to physical servers, virtualization technology can remap virtual machines and physical resources according to the change of load, so as to dynamically realize the load balance of the whole system. The remapping of virtual machine and physical resources is realized with the help of virtual machine dynamic migration technology. According to the characteristics of cloud computing platform, the goal of server virtualization computing resource scheduling is to automatically distribute the distribution of virtual computing resources on physical computing resources in a certain way, complete the integration of computing resources in cloud computing environment, and realize the on-demand allocation of computing resources and the dynamic expansion of resource pool. Its main functions include (1) resource allocation and recovery; (2) resource scheduling and optimization; and (3) system energy consumption and control. Realize resource allocation on demand, dynamic scaling of source pool, resource synchronization control, and automatic adjustment of resource distribution [20].

### 2.2. Structure Design of Cloud Platform Based on IoT

The smart community IoT platform uses new technologies to realize the functions of community environmental monitoring, home safety, and community/building monitoring, so as to provide a safe, healthy, and convenient living community for community residents [21, 22]. The smart community IOT platform realizes the centralized control and management of IOT terminals by connecting various sensors, cameras, access control, and fire smoke sensors in the community to the platform, so as to realize fast and efficient value-added service and management through intelligent means, and provide a safe and comfortable community living environment [23]. The smart community IoT platform is divided into three layers, namely terminal layer, network layer, and IoT management platform. Its architecture is shown in Figure 2.

The terminal layer of the intelligent community IoT platform is responsible for data collection to realize the monitoring of the community and community/family safety, while the network layer is responsible for the transmission of terminal data collection and control information. On the one hand, the Internet of things management platform stores and intelligently analyzes and processes the data collected from the device end. On the other hand, it provides authentication management function, device control function, and coordination of different terminal equipment functions, realizes the linkage between devices, enhances the unified management of Internet of things equipment in the community, and improves the comprehensive service level of the community.

The smart community applies 5G technology integration and Internet of things technology, which also enriches the means of ecological governance. In this process, the advantages of the two technologies can also be used to achieve the goal of unmanned monitoring. Whether it is environmental governance or environmental perception, the integration technology of the two can be used for network wide linkage, which also speeds up the pace of information construction, especially meets the accuracy of environmental monitoring and management. In order to promote the construction of community ecological environment, the community can also set up corresponding perceptual street lamps in the community and integrate the scattered contents to meet the construction needs of the system. In this process, it should also reserve pipelines, adjust according to the actual needs of the community, expand the electronic pile system, and realize energy conservation [24].

## 3. Research on Smart Community Big Data Dynamic Analysis Model Based on Logistic Regression Model

In order to minimize carbon emissions and maximize resource economy, the overall framework of the algorithm is designed in Figure 3. The algorithm framework mainly includes data sources, feature extraction, model training, data prediction, and result analysis visualization.

### 3.1. Research on Data Dimension Reduction Based on PCA Method

Smart community big data are difficult to be described in a unified way. However, if we only care about data collection and growth over time. Then, this kind of big data can be formatted as distributed data flow.

**Definition 1 .**

(Distributed data stream). Given time matrix *T*=〈*t*_1_, *t*_2_,…, *t*_*n*_〉, matrix dimension *d,* and IOT data acquisition node *n*, a distributed data stream is *S*={*S*_1_, *S*_2_,…, *S*_*n*_}, where each *S*_*k*_(*k*=1,2,…, *n*) is a multidimensional data tuple sequence collected on *S*_*k*_=〈*r*_1_, *r*_2_,…*r*_*t*_,…〉, *r*_*t*_=(*r*_*t*_^1^, *r*_*t*_^2^,…, *r*_*t*_^*d*^).

For the classified mining of big data with distribution and mobility, the data can be used as the collection model of training samples. For example, in systems such as network traffic monitoring and e-commerce transactions, this data model can be used to collect corresponding training data.  Figure 4 shows flow chart of distributed data mining.

At time point *t*, the task of classification mining is to use the time window at time *t* to update the local microcluster pattern and the global integrated classifier to the (current) state at time T, as shown in Figure 4, the classification mining of a big data has three relatively independent stages:

1. Local mining is to use the current data block chunk_*t*_ defined in Definition 1, and then chunk_*t*_ is implemented to incrementally increase the local microcluster pattern maintained by the previous mining point to form a new (current) microcluster pattern.
2. Pattern transmission. It mainly records the nodes that have been mined over time and update to the server.
3. Global mining. When collecting the mining nodes of all distributed servers, update the global status according to the latest requirements for the next step of distributed mining.

### 3.2. Research on Trace Detection and Detection of Abnormal Measurement Data

Assuming that there are *m* ≥ 1 receivers and the discrete data received by the *i*th nodes is *x*_*i*_(*n*),  *i*=1,2,…, *n*, there are the following two assumptions. (1) Suppose H0: only abnormal data, no valid data. (2) Hypothesis H1: there are both valid data and abnormal data.

The main diagonal element of the covariance matrix of measurement data is the embodiment of target data and abnormal data. When considering the existence and absence of effective data, respectively, there will be significant differences in the obtained trace function. By using the random matrix theory to analyse the trace function, a more accurate expression can be obtained in theory, and then the determination of the existence of the target can be realized.

Make *N*_*j*_=max(*N*_*ij*_), fill zero in other positions of *h*_*ij*_(*k*):

(1) $$\begin{array}{c} \left\{\begin{array}{c} x\left(n\right)=\left[x_{1}\left(n\right),x_{2}\left(n\right),\ldots ,x_{M}\left(n\right)\right],\\ h_{j}\left(n\right)=\left[h_{1j}\left(n\right),h_{2j}\left(n\right),\ldots ,h_{Mj}\left(n\right)\right],\\ \eta \left(n\right)=\left[\eta_{1}\left(n\right),\eta_{2}\left(n\right),\ldots ,\eta_{M}\left(n\right)\right]. \end{array}\right. \end{array}$$

For *L* outputs, define:

(2) $$\begin{array}{c} \left\{\begin{array}{c} \overset{⌢}{x}\left(n\right)=\left[x^{T}\left(n\right),x^{T}\left(n-1\right),\ldots ,x^{T}\left(n-L-1\right)\right],\\ \overset{⌢}{h}\left(n\right)=\left[h^{T}\left(n\right),h^{T}\left(n-1\right),\ldots ,h^{T}\left(n-L-1\right)\right],\\ \overset{⌢}{\eta }\left(n\right)=\left[\eta^{T}\left(n\right),\eta^{T}\left(n-1\right),\ldots ,\eta^{T}\left(n-L-1\right)\right]. \end{array}\right. \end{array}$$

The following functions are established according to the model:

(3) $$\begin{array}{c} \overset{⌢}{x}\left(n\right)=H\times s\left(n\right)+\overset{⌢}{\eta }. \end{array}$$

In equation (3), the diagonal element of the covariance matrix represents the sum of the energy projected by the effective data on each component. If there is abnormal data, the trace of the covariance matrix will change. The main diagonal element of the data covariance matrix is the embodiment of the effective data and abnormal data. When considering the existence and absence of effective data, respectively, the trace function obtained will be significantly different.

According to the random matrix theory, when only abnormal data are considered, the eigenvalue distribution of the covariance matrix of the measured data satisfies the M-P law, that is, all eigenvalues are concentrated in a ring, and the radius of the inner ring and the outer ring is deterministic quantities independent of the abnormal data. However, when the effective data exist, the large eigenvalues must fall on the outside of the ring. The target signal can be detected by analyzing the spectral distribution of eigenvalues. The law is embodied in the complex plane of the characteristic root, which is a ring with an inner circle radius of and an outer circle radius of 1.

### 3.3. Research on Prediction Algorithm Based on Logistic Regression Model

Logistic regression analysis is a generalized linear *r* model, which is utilized in data analysis fields. If the result of linear regression is a value and the value range cannot be limited, we can add function mapping by summing the feature linearly, calculate with function *g*(*z*), and map the continuous value to 0 or 1.

For a given *n* characteristics *x*=(*x*_1_, *x*_2_,…, *x*_*n*_), let the conditional probability of occurrence of observation sample *y* relative to event occurrence factor *x* be *p*(*y*=1*|x*) expressed by logistic function as

(4) $$\begin{array}{c} p\left(y=1|x\right)=\pi \left(x\right)=\frac{1}{1+e^{-g\left(x\right)}}, \end{array}$$

where function *g*(*x*)=*ω*_0_+*ω*_1_*x*_1_+⋯+*ω*_*n*_*x*_*n*_, then the probability that *y* does not occur under the condition of *x* is

(5) $$\begin{array}{c} p\left(y=0|x\right)=1-p\left(y=1|x\right)=\frac{1}{1+e^{g\left(x\right)}}. \end{array}$$

Assuming that there are *m* mutually independent observation events *y*=(*y*^(1)^, *y*^(2)^,…, *y*^(*m*)^), the occurrence probability of event (*y*^*i*^=1):

(6) $$\begin{array}{c} p\left(y^{i}\right)=p^{y^{\left(1\right)}}{\left(1-p\right)}^{1-y^{\left(i\right)}}. \end{array}$$

Then, for the whole data set, since each sample is independent of each other, the probability of *m* samples is multiplied by their respective probability of occurrence, and the likelihood function of *m* independent samples is:

(7) $$\begin{array}{c} L\left(\theta \right)=\prod_{i=1}^{m}f\left(x;\theta \right)={\prod_{i=1}^{m}\left(\pi \left(x\right)\right)}^{y^{\left(1\right)}}{\left(1-\pi \left(x\right)\right)}^{1-y^{\left(i\right)}}. \end{array}$$

In order to maximize *L*(*θ*), the purpose is to find the parameters *θ*_0_, *θ*_1_,…, *θ*_*n*_ and take logarithm of function *L*(*θ*) to obtain:

(8) $$\begin{array}{c} L\left(\theta \right)=\sum_{i=1}^{m}y^{\left(i\right)}\left(\theta^{T}x^{i}\right)-\sum_{i=1}^{m}\log\left(1+e^{\theta^{T}x^{\left(i\right)}}\right). \end{array}$$

The maximum likelihood *L*(*θ*) always calculated by gradient rise, and the solution value is the best parameter. Therefore, it can be multiplied by the negative coefficient −1/*m* and transformed into gradient descent method for solution, and then *L*(*θ*) is transformed into *J*(*θ*) as follows:

(9) $$\begin{array}{c} J\left(\theta \right)=-\frac{1}{m}L\left(\theta \right). \end{array}$$

## 4. Experiment and Result Analysis

Data sources: it is a sample in a city, which adopts multistage and hierarchical sampling, and selects 100 elderly people over the age of 65 in five communities as the survey objects. The reason why the region is selected as the research sample is that one of the regions with serious aging in a city has a large elderly population, which is more conducive to the research. Songjiang District has an obvious trend of population aging. Therefore, the samples collected in this area have an objective and comprehensive response to the elderly care services combined with smart communities to be investigated in this paper.

The features selected for modelling are briefly described. The feature set is divided into five categories: basic family situation, education, health status, income and expenditure characteristics, and life safety. In terms of the basic situation of families, it mainly includes the situation of migrant workers, power supply, the number of family dropouts due to poverty, etc. From the analysis of family education, education level and the status of students in school have a positive correlation in the life happiness index. Family education level has a potential impact on personal quality and children's education, and there are different differences in adapting to society. From the perspective of family health status and life safety, health status will affect family income, family life burden, children dropping out of school, and so on. From the analysis of the characteristics of family income and expenditure, the nature of family income includes various state subsidies and property income. The above feature selection shows that the research on the aging population in China is very complex. Comprehensively read the relevant literature and generally determine the above attributes as the characteristics of the smart community prediction model through the above experiments.

Simulation environment: in order to simulate distributed big data, we have developed a software tool stream producer to produce data flow. It simulates the online arrival of flow data through I/O operation of KDD99 data set. This experiment is based on four Intel Core i7 computer with 2 GB memory.

### 4.1. Analysis of Data Anomaly Detection and Spectral Distribution

The Internet of things has a large amount of data, high dimension, complex relationship, strong relevance, and specialty. It belongs to the typical application field of industrial big data. It reflects the track information, performance changes, working mode switching, and failure of the Internet of things and provides an effective basis for effective analysis and intelligent calculation of Internet of things data and various operation, maintenance, and management work. It is different from the change law of normal Internet of things data, which can reflect the failure of acquisition equipment, damage of transmission link, performance degradation of corresponding equipment, quality problems, mechanical and electronic faults, or insufficient design. Timely and effectively discover the abnormal patterns in the Internet of things data and carry out remote command repair, transmission link repair, software troubleshooting, fault plan formulation, or maintenance service optimization for the tested equipment, which has significant practical significance for improving the ground service quality and enhancing the maturity, security, and reliability of all links of Internet of things design, development, production, and maintenance.

Figure 5 shows the trace curve of abnormal data in case of large interference, small interference, and no interference. When the system operates normally, the trace curve is close to a straight line, and its slope change rate is close to 0, that is, there is no abnormal data; when the system is disturbed, the trace curve has obvious bending changes, and the changes of the curve are different when different disturbances occur. The change of large disturbance curve is more obvious than that of small disturbance curve, and the change rate of curve slope is also faster. Through the comparison of the three curves, it is found that the change degree of the curve has an obvious strong correlation with whether the system has disturbance and the size of disturbance. Therefore, the occurrence of system disturbance can be judged through the abnormal data detection of matrix trace. The fault start time is 0.1 s, and the fault removal time is 0.2 s. Collect PMU data 5 s after the fault occurs. The spectrum analysis results of the three simulations are shown in Figure 6, in which the distribution points in the ring are the normal data of the system and the distribution points in the inner ring are the abnormal data.

When the system operates normally, there is no fault, there are almost no abnormal data points in the inner ring area, and there are a small number of distribution points at the edge of the inner ring. The calculation and analysis results show that these error points account for about 2.5% of the total data points. The main reason is the system error and other factors, which have no interference on the abnormal detection and judgment. When the fault set in the simulation occurs, abnormal data points begin to appear in the inner ring area, and the number of distribution points in the inner ring will obviously change with the fault type and the interference of the system, as is shown in Figure 6(a). Among them, in case of small interference fault, as shown in Figure 6(b), some inner ring distribution points appear. According to the analysis of calculation results, the proportion of all distribution points is about 12%. In case of large disturbance fault in the system, Figure 6(c) shows that there are many distribution points in the inner ring, accounting for about 35% of all distribution points.

From the above analysis, it can be found that in the big data modeled by high-dimensional random matrix, the abnormal data generated by different disturbances of the system can be detected by spectral analysis, and its change law can be seen. To sum up, when the system operates stably and fails, the proportion of abnormal data detected by this method changes significantly; with the increase of system fault severity, the proportion of abnormal data increases and the order of data distribution decreases.

### 4.2. Efficiency Verification of Distributed Data Mining

In order to verify the efficiency of distributed data mining, we control several other parameters unchanged. The improved BDS scheme is compared with BDS scheme in the data flow within 500 s. Then, collection data in KDD99 are used for validation.  Figure 7 shows the change of error rate of two schemes with the increase of history data length.

This experiment is based on a distributed data flow application environment with three local nodes and one central node. Four Intel Core i7 computers with 2 GB memory are used to form the corresponding hardware unit. Using Hadoop's HDFS distributed file system, KDD99 data sets are distributed and stored in three local nodes, and the central node is used as the master node. Responsible for maintaining the corresponding file directory information, on each local node, the stream producer tool is deployed to simulate the generation process of data flow to form window data.

Figure 7 shows that the error rate of improved BDS is significantly lower than that of BDS (better than about 10% on average).  Figure 7 shows that the accuracy of improved BDS is gradually improved, and BDS shows fluctuation. So it is impossible to exchange the classification accuracy by infinitely increasing the window length. In addition, compared with BDS, the accuracy stability of improved BDS is better. As far as Figure 7 is concerned, when the window length reaches 30 s, the error rate of improved BDS keep balanced and keep at 13%. The continuous increase of time window cannot bring the decrease of error rate.

Execute improved BDS and BDS once every 100 s to 500 s and then test the accuracy.  Figure 8(a) shows the change of the error rate of improved BDS under different numbers of weak classifiers (the comparison algorithm is BDS). In addition, in order to see the difference between the two methods more clearly, Figure 8(b) shows the error rates of improved BDS and BDS under different running environment. The simulation results show that the improved BDS scheme is obviously better than the conventional BDS scheme. When the ensemble classifier maintains a certain number of weak classifiers (e-NO = 20 in the experiment), the classification accuracy of BDS ensemble will gradually improve with the increase of training time and gradually stabilize within a certain accuracy range. In contrast, DS means has a certain fluctuation.

### 4.3. Comparison Results Analysis

The effectiveness of this study is the same in 10 communities. Five were selected as the control group and five as the experiment group. The control group was carried out according to the original construction plan, and the experimental group adopted the construction of smart community. Observe and study from six indicators: service efficiency, service evaluation, prediction accuracy, construction planning, construction standard, and intellectualization.  Table 1 records the change trend of the control group and the experiment group in 18 months.

Table 1 shows that with the increase of time, the indexes of the control group did not increase significantly; the experimental group basically kept a balance with the control group in the first six months. After the transformation in December, various indicators increased significantly, especially the degree of intelligence was greatly improved. The comparison results can verify the reliability and superiority of the scheme.

## 5. Conclusion

This paper first analyses and introduces the problems and development trends existing in the development of domestic smart communities and analyses the needs of smart community construction from three aspects: basic needs, functional needs, and performance needs, then studies and analyses the key technologies involved in the process of smart community construction, and finally designs the overall design of the whole smart home integrated service management platform on this basis. Second, aiming at the abnormal data in high-dimensional data, an abnormal measurement data detection method based on random matrix theory is proposed. In the process of anomaly detection, through trace detection and spectral distribution detection in random matrix theory, the measured data can be analysed theoretically to realize the detection of targets (measured abnormal data); finally, a prediction scheme based on logistic regression model is designed. Simulation results verify the effectiveness and reliability of the scheme. In general, aiming at the shortcomings of low informatization of domestic communities and less application of IoT, this paper integrates the functional and performance needs of residents for the living environment and puts forward a smart community construction scheme based on IoT to meet the living needs of community residents. This scheme has strong reproducibility, is suitable for most regions, and has practical guiding value in the construction of smart communities. Further work includes for the non-normal data distribution, the sample reconstruction method based on density estimation is studied; find the global pattern mining method of nonsample reconstruction technology; for other needs of big data, research mining problems other than classification, such as association rules and concept induction; according to other technical characteristics of big data, such as high dimensionality and semi-structured data, research on corresponding theories, models, and algorithms is carried out.

## Figures and Tables

**Figure 1:** System architecture design based on IoT.

**Figure 2:** Architecture figure of smart community IoT platform.

**Figure 3:** Overall structure figure of algorithm.

**Figure 4:** The schematic figure for distributed and streaming big data mining.

**Figure 5:** Trace distribution of different state system.

**Figure 6:** Abnormal data distribution map under different conditions. (a) Distribution diagram without interference, (b) distribution diagram under small interference, and (c) distribution diagram with big interference.

**Figure 7:** Change of error rate under different lengths of time window.

**Figure 8:** Simulation results and analysis. (a) Change of error rate of mobile data and (b) error rate under same parameters.

**Table 1:** Comparison results analysis.

Indicators	6 months		12 months		18 months	
	Control group	Experiment group.	Control group	Experiment group.	Control group	Experiment group.
Service efficiency	51.3	50.5	58.6	51.2	72.6	52.3
Service evaluation	48.6	48.3	52.4	48.2	70.3	49.1
Prediction accuracy	77.1	76.9	80.5	77.1	89.6	77.5
Construction planning	68.4	69.7	72.1	70.0	79.2	71.6
Construction standard	54.6	55.3	61.2	56.4	63.4	58.9
Intellectualization	36.5	31.4	50.7	33.6	80.6	36.7

## Data Availability

The data used to support the findings of this study are available from the corresponding author upon request.
